The article "Diagnosis of Schizophrenia Based on Deep Learning Using fMRI" was published in 2021. Journal: Comput Math Methods Med.

# Diagnosis of Schizophrenia Based on Deep Learning Using fMRI

**DOI:** 10.1155/2021/8437260

**Published:** 2021-11-09

**Authors:** JinChi Zheng, XiaoLan Wei, JinYi Wang, HuaSong Lin, HongRun Pan, YuQing Shi

**Affiliations:** ^1^Quanzhou Third Hospital, Quanzhou 362000, China; ^2^Quanzhou First Hospital Affiliated to Fujian Medical University Neurology Department, Fujian, China; ^3^The Second Affiliated Hospital of Fujian Medical University Neurology Department, Fujian, China; ^4^Jinjiang Third Hospital, Quanzhou 362000, China

## Abstract

Schizophrenia is a brain disease that frequently occurs in young people. Early diagnosis and treatment can reduce family burdens and reduce social costs. There is no objective evaluation index for schizophrenia. In order to improve the classification effect of traditional classification methods on magnetic resonance data, a method of classification of functional magnetic resonance imaging data is proposed in conjunction with the convolutional neural network algorithm. We take functional magnetic resonance imaging (fMRI) data for schizophrenia as an example, to extract effective time series from preprocessed fMRI data, and perform correlation analysis on regions of interest, using transfer learning and VGG16 net, and the functional connection between schizophrenia and healthy controls is classified. Experimental results show that the classification accuracy of fMRI based on VGG16 is up to 84.3%. On the one hand, it can improve the early diagnosis of schizophrenia, and on the other hand, it can solve the classification problem of small samples and high-dimensional data and effectively improve the generalization ability of deep learning models.

## 1. Introduction

Schizophrenia is a serious and disabling mental illness. It is manifested as obstacles such as thinking, emotion, and behavior, the condition shows a slow and progressive development, and there are various degrees of social function defects. Symptoms include false beliefs, unclear or confused thinking, hearing voices that others cannot hear, reduced social participation and emotional expression, and lack of motivation. It not only brings great pain to the patient, but also a heavy burden to the family and society. It is about 1% of the diseased population worldwide [1]. Early diagnosis and effective intervention and treatment of schizophrenia can improve the disease. The cure rate is to prevent the prolonged course of the disease. However, the etiology and pathogenesis of schizophrenia are still unclear, and objective laboratory diagnostic indicators, as well as diagnostic criteria for equipment, are lacking. The clinical diagnosis is mainly based on medical history, combined with psychiatric symptoms and the law of progression of the disease and scales. Due to the complexity of the pathological mechanism, the early diagnosis of schizophrenia is still a challenging problem. Schizophrenia has a serious negative impact on human perception, thinking, emotion, and behavior, and it mostly occurs in people aged 15 to 34. This disease has the characteristics of early controllable, late recurrent attacks, and severely impaired cognitive function [2].

At present, the diagnosis of schizophrenia is mainly based on the patient's behavior, such as the commonly used positive and negative symptom scales for quantitative evaluation [3]. The clinical diagnosis of patients is mainly based on the doctor's experience and related scale evaluations, and there is a lack of objective diagnostic criteria. Some studies have even found that after effective treatment, the level of inflammatory factors in patients with schizophrenia will decrease significantly. IL-6 may be the most important cytokine involved in the inflammatory response. IL-8 is a member of the chemokine family. Previous studies have found that both are positively correlated with negative symptoms of schizophrenia [4]. Other scholars have found that IL-1*β* gene expression level is positively correlated with PANSS general psychopathological symptoms, and serum IL-1*β* of patients with schizophrenia is significantly positively correlated with PANSS total score. As a multifunctional proinflammatory factor, TNF-*α* has been found to be negatively correlated with the total score of PANSS and the score of general psychopathological symptoms in patients with chronic schizophrenia. It is suggested that the level of the abovementioned proinflammatory factors may be related to the symptoms of schizophrenia patients. However, it may be affected by confounding factors such as small sample size and failure to control substance use. Due to the complexity of the correlation between schizophrenia and inflammatory factors and the subjectivity of the doctor's diagnosis, missed and misdiagnosed situations may occur. Therefore, there is an urgent need to develop an effective computer-aided diagnosis system to assist doctors in achieving accurate diagnosis of schizophrenia.

With the rapid development of science and technology, with the implementation of deep learning [5], computer-aided diagnosis has been widely used in brain structure functional magnetic resonance image, fMRI research, such as brain tumor segmentation [6–8], Alzheimer's disease classification [9–11], and ADHD diagnosis [12–14]; it also provides an effective method for the classification of schizophrenia.

Between 2014 and 2018, more than 55% of neuroimaging studies of brain diseases used support vector machine (SVM) [15]. Lu et al. [16] proposed schizophrenia as MRI study calculated the gray matter and white matter volumes of each brain region of interest (ROI) and took the significant difference between the two as input features and used SVM classification. Liu et al. [17] constructed a hierarchical brain network by measuring the cortical thickness of each ROI of the brain, extracting the node and edge features of the network, and inputting it into the SVM to realize the auxiliary diagnosis of schizophrenia. Huang et al. use the mathematical tool Pearson's correlation coefficient to calculate the correlation coefficient between fMRI brain regions, and the features after dimensionality reduction by principal component analysis are used for SVM learning. Yang et al. used three methods to analyze fMRI images to obtain three fMRI features, and the three features were used to train three capsule neural networks. Finally, the classification result is obtained through the method of ensemble learning. Yang et al. input the functional connection coefficients after PCA dimensionality reduction as features into the neural network to obtain a classification model.

At present, some reviews have summarized and analyzed the application of deep learning [18–21] in the field of medical imaging [22]. However, there is no literature to systematically sort out and summarize the deep learning methods based on magnetic resonance imaging used in the diagnosis of schizophrenia. In view of this, this article will start from the perspective of deep learning and use VGG16 to extract effective information from fMRI data to diagnose patients with schizophrenia.

## 2. Methodology

### 2.1. VGG16

The convolutional neural network (CNN) [22] is shown in Figure 1, which includes a convolutional layer, a downsampling layer, and a fully connected layer. Each layer has multiple feature maps, and each feature map has multiple neurons, and the input features are extracted through the convolution filter [23]. The parameter sharing mechanism of the convolutional layer greatly reduces the number of parameters [24].

The research is based on the VGG16 network to optimize and improve the network. The main structure of VGG16 [16] consists of 5 convolution modules, 3 fully connected layers, and an input layer and output layer. Each convolution layer module is downsampled through max pool.

The expression of the convolutional layer is as follows:

(1) $$\begin{array}{c} x_{j}^{l}=f\left(\underset{i\in M_{J}}{\sum }x_{i}^{l-1}*k_{ij}^{l}+b_{j}^{l}\right). \end{array}$$

In Equation (1), assuming that *l* − 1 is the input layer or the pooling layer, and the *l* layer is the convolutional layer, then *x*_*i*_^*l*^ is the *j*-th feature map of the *l* convolutional layer; the right side of Equation (1) represents the feature map of the *l* − 1 layer. Perform convolution operation with the *j*-th convolution kernel *k*_*ij*_^*l*^ of the l layer and sum; *b* represents the bias; *f*(·) is the activation function ReLU.

The pooling layer closely follows the convolutional layer and plays the role of scaling dimensionality. The calculation equation is as follows:

(2) $$\begin{array}{c} x_{i}^{l}=f\left(\beta_{j}^{l}\text{down}\left(x_{i}^{l-1}\right)+b_{j}^{l}\right). \end{array}$$

In Equation (2), down(·) is the pooling function, which seeks the maximum value for a region of the feature map; *β*_*j*_^*l*^ and *b*_*j*_^*l*^, respectively, represent the weight and bias of pooling.

The input layer size of VGG16 is 224 × 224 × 3, and the convolution module is composed of a stack of convolution layers and pooling layers. The convolution kernel is usually 3 × 3 with a step size of 1, and the pooling layer is a 2 × 2 max pool. Using the convolutional layer and the pooling layer to cooperate, on the one hand, the image size is reduced and the amount of model calculation is controlled. On the other hand, the convolution data of the large receptive field is obtained indirectly, and the high-dimensional feature map is obtained. The convolution module is followed by three fully connected layers to obtain the classification information of the feature map, and finally, the softmax layer is used to output the classification results. The structure diagram of the VGG16 network is shown in Figure 2.

The increase in the depth of the convolutional neural network in the VGG16 network and the use of small convolution kernels have a great impact on the final classification and recognition effect of the network. The convolutional layers all use the same 3-size convolution kernel parameters, and the pooling layers all use the same pooling kernel parameters. The combination of multiple 3 × 3 convolutional layers not only has a small amount of calculation, but also obtains the same receptive field of the large convolution kernel at the same time. The deep network structure verifies the conjecture that network performance can be improved by continuously deepening the network structure. But for some data, a too deep network only greatly increases the training time, but does not improve the accuracy. The convolution kernel of VGG16 increases from 64 to 512 sequentially, and the number of image channels is first reduced to 64 and then increased to 512. However, due to the large amount of image data, this change in the number of channels will cause the data to lose a lot of information. Increasing the time cost of training and the network structure of VGG16 for this research task, while increasing the depth of the network, cannot improve the accuracy of the network.

### 2.2. Improved VGG16 Model

Convolutional neural networks are mainly composed of convolutional layers, nonlinear units, pooling layers, and fully connected layers. In the classification problem, the convolutional layer, the nonlinear unit, and the pooling layer are used as the feature extraction layer to extract features, and the fully connected layer is used as the classification layer for classification. The convolutional layer is the core of the convolutional neural network, and the convolution equation is shown in Equation (3).

(3) $$\begin{array}{c} y\left(t\right)=\int_{-\infty }^{\infty }x\left(p\right)h\left(t-p\right)dp=x\left(t\right)\times h\left(t\right). \end{array}$$

The nonlinear unit is the ReLU activation function, and its expression is shown in Equation (4).

(4) $$\begin{array}{c} y=\max\left(0,x\right). \end{array}$$

The pooling layer is a downsampling operation to reduce the dimensionality of the extracted features while retaining important information of the features.

The VGG16 network is trained on a large data set ImageNet. The ImageNet data set is a 1000 classification problem data set, so the classification layer parameters of the VGG16 network are huge. The diagnosis of schizophrenia is a two-class classification problem and does not require a complex classification layer. Therefore, the feature extraction layer of the VGG16 network is retained, the classification layer is redesigned, and the original 3-layer fully connected layer is improved to a 2-layer fully connected layer. We take the features of 3 convolutional layers and 3 pooling layers as an example, and the process of part of the extracted features is shown in Figure 3. Use the ReLU activation function, and add a dropout layer to prevent overfitting, and change the final output classification to two categories. The data can be divided into schizophrenia and nonschizophrenia, and the amount of parameters is reduced, so that the network converges faster, and the recognition speed of the data is improved.  Figure 4 shows the improved VGG16 schizophrenia classification model.

### 2.3. Transfer Learning

Transfer learning solves the shortcomings of deep learning that requires a large number of sample training models. By training a pretrained model on a large data set, it is possible to use a small number of data sets to train the model. Fine-tune is a training method that retains the model feature extraction layer and retrains the model classification layer. The pretraining model used is the VGG16 network pretrained on the ImageNet data set, and the feature extraction layer of the pretraining model is fixed. Retrain the improved classification layer of VGG16 to complete the training of the schizophrenia classification model.  Figure 5 shows the transfer learning training process.

## 3. Results

### 3.1. Data Set

This experimental data set comes from the public data set of the Center for Biomedical Research Excellence (COBRE). The address of the COBRE data set is http://fcon_1000.Projects.nitrc.org/indi/retro/cobre.html. The data set in this paper contains 200 samples between the ages of 18 and 65. The information is shown in Table 1. In this paper, the original data is preprocessed by binarization, standardization, and smoothing. The specific process is shown in Figure 6.

### 3.2. Evaluation Index

We use evaluation indicators commonly used in classification tasks: precision, recall, accuracy, and AUC.  Table 2 illustrates the classification task through the confusion matrix. True positive (TP) indicates that the positive class is predicted as a positive class, and the number of sample positive classes was actually predicted by the model. False negative indicates (FN) that the positive class is predicted as a negative class, and the number of negative classes in the sample was actually predicted by the model. False positive (FP) indicates that the negative class is predicted as a positive class, and the number of positive classes of samples was actually predicted by the model. True negative (TN) indicates that the negative class is predicted as a negative class, and the number of sample negative classes was actually predicted by the model.

*The definition of recall rate*: it is the proportion of the true correct accounted for all actual positive. The calculation equation is as follows.

(5) $$\begin{array}{c} \text{Recall}=\frac{\text{TP}}{\text{TP}+\text{FN}}. \end{array}$$

*The definition of accuracy*: it is the proportion of all predictions that are truly correct. The calculation equation is as follows.

(6) $$\begin{array}{c} \text{Precision}=\frac{\text{TP}}{\text{TP}+\text{FP}}. \end{array}$$

### 3.3. Model Comparison

The algorithm under study is implemented on the deep learning framework TensorFlow and PyTorch platform and is programmed in Python language. The experiment did a detailed study on the schizophrenia recognition rate, accuracy rate, recall rate, and area under curve (AUC). The framework proposed by the research uses the COBRE data set. In order to further verify the effectiveness and superiority of the model proposed in this research, the test set is compared with the existing mainstream framework models.  Table 3 gives the results of the evaluation indicators of different models. It can be seen that the framework proposed in this study has the highest classification accuracy rate (87.85%) and the highest accuracy rate (87.11%) compared with the current several popular methods. And the highest recall rate is 89.63%. The diagnostic accuracy rates of AlexNet, VGG16, and ResNet50 models are 78.36%, 85.27%, and 83.09%, respectively. It shows that the proposed schizophrenia diagnosis network is better than other comparison models in accuracy, precision, and recall and can effectively complete the classification task. The receiver operating characteristic (ROC) curves of the four models are shown in Figure 7. Unlike other network models, the accuracy and recall rates of our proposed network model are relatively balanced. At the same time, the AUC index of our proposed model is also higher than that of other models, which proves our model that can learn the essential feature of the data. The generalization ability of the model is better.

## 4. Discussion

In this study, the diagnosis model of schizophrenia patients and normal people is based on the deep learning algorithm of fMRI data. Schizophrenia is a very serious mental disorder. At present, it is diagnosed clinically based on the corresponding diagnostic scale and doctor's experience, mainly based on the progress of the disease. This study uses objective EEG data and uses deep learning algorithms to establish a mathematical model for differential diagnosis of the disease, and good results have been achieved.

It can provide a reference for clinical diagnosis and improve the diagnosis ability of clinicians for schizophrenia so as to find the condition in time and give timely treatment.

In order to solve the problems of low accuracy in pathological recognition and complex feature engineering construction in traditional artificial recognition, a schizophrenia diagnosis model based on convolutional neural network algorithm was constructed through deep learning. The network first uses VGG16 for migration learning, then extracts the features of fMRI by designing the convolution structure of the neural network, and finally uses the fully connected layer for training and continuous optimization to obtain the optimal weight parameters.

Finally, the recognition of schizophrenia diagnosis can be achieved. The proposed model has a strong characterization ability for data features and achieved an accuracy of 87.85% in COBRE, which is 2.31 percentage points higher than the existing VGG16 algorithm. Further improvements are needed to meet actual application requirements. It has good application prospects. The application of deep learning in the diagnosis of schizophrenia based on magnetic resonance imaging is a research direction with both challenges and opportunities. In order to promote the transformation of deep learning models from the research stage to practical applications, researchers still need to conduct more systematic and in-depth exploration.

## Figures and Tables

**Figure 1:** Convolutional neural network structure.

**Figure 2:** VGG16 structure.

**Figure 3:** Feature visualization.

**Figure 4:** The improved VGG16 schizophrenia classification model.

**Figure 5:** Transfer learning training process.

**Figure 6:** Data preprocessing process.

**Figure 7:** The ROC curves of the four models.

**Table 1:** Participant information.

Category	Healthy	Sick	*P* value
Number of people	102	98	
Average age (standard deviation)	36.85 (11.86)	37.46 (12.99)	0.55
Gender (male/female)	55/47	59/39	

**Table 2:** Confusion matrix.

Data type	Predicted positive class	Predicted negative class
Actual positive class	TP	FN
Actual negative class	FP	TN

**Table 3:** Comparison of effects of different models.

Different models	Accuracy	Precision	Recall	AUC
AlexNet	78.36%	81.29%	75.66%	0.76
VGG16	85.27%	86.33%	87.48%	0.83
ResNet	83.09%	86.59%	79.98%	0.81
Our model	87.58%	87.11%	89.63%	0.85

## Data Availability

The image data used to support the findings of this study have been deposited in the Center for Biomedical Research Excellence (COBRE) data set (http://fcon_1000.Projects.nitrc.org/indi/retro/cobre.html).
